# First Report of *Vibrio tubiashii* Associated with a Massive Larval Mortality Event in a Commercial Hatchery of Scallop *Argopecten purpuratus* in Chile

This article has been retracted.

**DOI:** 10.3389/fmicb.2016.01473

**Published:** 2016-09-20

**Authors:** Rodrigo Rojas, Claudio D. Miranda, Javier Santander, Jaime Romero

**Affiliations:** ^1^Laboratorio de Biotecnología, Instituto de Nutrición y Tecnología de los Alimentos, Universidad de ChileSantiago, Chile; ^2^Laboratorio de Patobiología Acuática, Departamento de Acuicultura, Universidad Católica del NorteCoquimbo, Chile; ^3^Centro AquapacíficoCoquimbo, Chile; ^4^Laboratorio de Patogénesis Microbiana y Vacunación, Facultad de Ciencias, Universidad MayorSantiago, Chile

**Keywords:** *Vibrio tubiashii*, *Scallop larvae*, Vibriosis, Shellfish pathology, Argopecten purpuratus

## Abstract

The VPAP30 strain was isolated as the highly predominant bacteria from an episode of massive larval mortality occurring in a commercial culture of the Chilean scallop *Argopecten purpuratus*. The main aims of this study were, to characterize and identify the pathogenic strain using biochemical and molecular methods to demonstrate its pathogenic activity on scallop larvae, to characterize its pathogenic properties and to describe the chronology of this pathology. The pathogenic strain was identified as *Vibrio tubiashii* based on its phenotypic properties and the sequence analysis of its 16S rRNA and housekeeping genes (*ftsZ, gapA, gyrB, mreB, pyrH, recA, rpoA* and *topA*). When triplicate cultures of healthy 10*–*day*–*old scallop larvae were challenged with 1 × 10^5^ colony forming units (CFU) mL^-1^ of the VPAP30 strain, percentages of larval survival of 78.87 ± 3.33%, 34.32 ± 4.94%, and 0% were observed at 12, 24, and 36 h, respectively; whereas uninfected larval cultures showed survival rates of 97.4 ± 1.24% after of 48 h. Clinical symptoms exhibited by the scallop larvae infected with the VPAP30 strain include the accumulation of bacteria around the scallop larvae, velum disruption and necrosis of digestive gland. The 50% lethal dose (LD_50_) of VPAP30 strain at 24 and 48 h was 1.3 × 10^4^ and 1.2 × 10^3^ CFU mL^-1^, respectively. The invasive pathogenic activity of the VPAP30 strain was investigated with staining of the bacterial pathogen with 5-DTAF and analyzing bacterial invasion using epifluorescence, and a complete bacterial dissemination inside the larvae at 24 h post-infection was observed. When scallop larvae were inoculated with cell-free extracellular products (ECPs) of VPAP30, the larval survival rate was 59.5 ± 1.66%, significantly (*P* < 0.001) lower than the control group (97.4 ± 1.20%) whereas larvae treated with heat-treated ECPs exhibited a survival rate of 61.6 ± 1.84% after 48 h of exposure. This is the first report of the isolation of *V*. *tubiashii* from the diseased larvae of the scallop *A*. *purpuratus*, occurring in a commercial culture in Chile, and it was demonstrated that the VPAP30 strain exhibits high pathogenic activity on scallop larvae, mediated both by bacterial invasion and the production of toxigenic heat-stable compounds.

## Introduction

The culture of the Chilean scallop *Argopecten purpuratus* (Lamarck, 1819) is the second most important industry in Chilean mariculture and is primarily concentrated in the north region of the country (von Brand et al., 2006); however, recurrent episodes of larval mortalities mainly due to bacterial infections have been observed, causing high economical losses and consequently precluding the sustainability of this industry. These bacterial infections are commonly characterized by a sudden cessation of larval motility leading to massive mortalities of reared larvae. Previous studies demonstrated the pathogenic activity of bacterial strains identified as *Halomonas* sp. (Rojas et al., 2009), *Vibrio anguillarum*-related (Riquelme et al., 1995), *Vibrio splendidus* (Rojas et al., 2015a) and the association of *Aeromonas hydrophila* and *Vibrio alginolyticus* (Riquelme et al., 1996) on scallop larvae.

*Vibrio* species have been described worldwide as the main aetiological agents of bacterial pathologies affecting reared larvae of various shellfish species (Waechter et al., 2002; Anguiano-Beltrán et al., 2004; Estes et al., 2004; Gay et al., 2004; Gómez-León et al., 2005; Prado et al., 2005, 2014, 2015; Labreuche et al., 2006; Garnier et al., 2007; Rojas et al., 2015a; Dubert et al., 2016b). Clinical symptoms commonly exhibited by reared shellfish larvae affected by vibriosis include the reduction of larval motility, erratic swimming, closing of valves, velum detachment, and bacterial swarming inside and around the larvae (Prado et al., 2005; Beaz-Hidalgo et al., 2010; Rojas et al., 2015a). Most of these clinical signs were described in larval cultures of the clam species *Ruditapes decussatus* (Gómez-León et al., 2005) and *Ruditapes philippinarum* (Dubert et al., 2016a), oyster species *Crassostrea virginica* (Gómez-León et al., 2008) and *Crassostrea gigas* (Estes et al., 2004; Gay et al., 2004; Garnier et al., 2007; Elston et al., 2008), and scallop species *Pecten maximus* (Nicolas et al., 1996; Torkildsen et al., 2005), *Argopecten ventricosus* (Sainz et al., 1998; Luna-González et al., 2002) and *Patinopecten yessoensis* (Liu et al., 2013). The pathogenicity of *Vibrio* strains causing vibriosis outbreaks is mediated by bacterial invasion (Rojas et al., 2015a; Dubert et al., 2016a) as well as the production of toxigenic extracellular products (ECPs) (Elston and Leibovitz, 1980; Labreuche et al., 2006; Binesse et al., 2008; Hasegawa et al., 2008; Labreuche et al., 2010; Rojas et al., 2015a).

*Vibrio tubiashii* was recognized 50 years ago as an important pathogen of hard clam and oyster larvae (Tubiash et al., 1965, 1970), causing the pathology “bacillary necrosis”, characterized by disruption and loss of cilia of the larval velar apparatus, high bacterial colonization of the larval shell and mantle, and abnormal swimming behavior. Later, Elston et al. (2008) reported a re-emergence of vibriosis episodes caused by *V*. *tubiashii* in a shellfish hatchery in North America producing an important loss of the intensive production of Pacific (*Crassostrea gigas*) and Kumamoto (*C*. *sikamea*) oysters and the geoduck clam *Panope abrupta*. However, this may be controversial because more recent studies re-classified (Wilson et al., 2013; Richards et al., 2014) some of these pathogenic strains as *V. coralliilyticus*, as well as other bivalve pathogenic *Vibrio* strains previously identified as *V. tubiashii* (Hada et al., 1984; Estes et al., 2004), demonstrating a high genomic similarity between both species (Ben-Haim et al., 2003; Ushijima et al., 2014).

Despite that efficient rearing techniques for scallop larvae production that have been developed, Chilean commercial hatcheries are currently suffering recurrent episodes of high mortalities of reared larvae, mainly associated with high levels of vibrio (Miranda et al., 2014; Rojas et al., 2015a). The identification of bacterial strains causing epizootics in larval cultures and understanding their pathogenic activity are essential for the development of adequate and efficient protocols of larval management, as well as for implementing proper bacteriologic monitoring strategies to prevent and control bacterial outbreaks occurring in commercial hatcheries of scallop larvae.

Considering that knowledge of the identity and pathogenic mechanisms of bacterial pathogens causing massive mortalities of scallop larvae reared in commercial hatcheries in Chile remains scarce, the aims of this study were to characterize and identify a highly pathogenic *Vibrio* strain recovered from massive larval mortality event that occurred in a commercial hatchery, to characterize its pathogenic properties and to describe the chronology of the pathology.

## Materials and Methods

### Bacterial Isolation

The pathogenic strain VPAP30 was recovered from a massive mortality event of reared-larvae of the scallop *A*. *purpuratus* occurring in a commercial hatchery located in Tongoy Bay in the north of Chile. Triplicate samples of settled dead and moribund larvae were aseptically collected from the bottom of the rearing tank during its water exchange using a sterile glass flask and were transported to the laboratory for immediate processing. Larval samples were centrifuged at 960 g for 2 min using an Eppendorf Model 5415D centrifuge (Hamburg, Germany) and the water excess was discarded. Settled larvae were ground by hand using a sterile glass digester containing 2 mL of sterile physiological saline (0.85% NaCl; PS) to obtain a homogenate according to the method of Nicolas et al. (1996). The homogenate was inoculated in triplicate onto Tryptic Soy Agar (Difco, NJ, USA) with 2% of NaCl (Oxoid, Hants, UK) (TSA2), and plates were incubated at 20°C for 48 h. The predominant colony grown almost as a pure culture in plates seeded with triplicate larval samples was isolated using TSA2 and the bacterial strain was preserved at -85°C in CryoBank (Mast Diagnostic, Merseyside, UK) vials prior use.

### Biochemical and Physiological Characterization

The phenotypic characteristics suggested by Noguerola and Blanch (2008) to identify *Vibrio* species, including cell morphology, Gram stain, oxidation/fermentation of glucose, and resistance to the vibriostatic agent O129 (2,4-diamino-6,7-diisopropylpteridine) (10 and 150 μg per disk) were determined according to the protocols described in Barrow and Feltham (1993). In addition, other phenotypic properties of VPAP30 strain were determined. Production of luminescence was detected in absence of light by using Marine agar 2216, whereas β-haemolysis of red cells was determined by using Columbia Blood agar (Oxoid, Hants, UK). Production of Møller’s lysine and ornithine decarboxylases and Thornley’s arginine dihydrolase were detected according to Hansen and Sörheim (1991). Growth at 4, 20, 30, 35, and 40°C was tested on Tryptic Soy broth supplemented with 2% NaCl (TSB2) and growth at 0, 3, 6, 8, and 10% of NaCl was assayed using peptone broth (BD, Sparks, USA). Additional phenotypic characteristics of VPAP30 strain were determined by using the API 20E (bioMérieux, Marcy-l’Etoile, France) and the Biolog (Biolog Inc., Hayward, CA, USA) systems. For the API system the VPAP30 strain was inoculated according to the manufacturer’s instructions with the modifications suggested by MacDonnell et al. (1982) and the API strip was incubated at 20°C for 48 h. For the Biolog system the strain was inoculated by using a solution containing 2.5% NaCl, 0.8% MgCl_2_, and 0.05% KCl, according to the instructions of the manufacturer and the microplate was aerobically incubated in the dark at 20°C for 72 h. For the API 20E and Biolog multi-inoculation tests, readings were made after 48 and 72 h of incubation, respectively.

### Enzymatic Analysis

The enzymatic activities of VPAP30 strain were determined by using the API ZYM system (bioMérieux, Marcy-l’Etoile, France) according to the manufacturer’s guidelines. Briefly, VPAP30 strain was cultured overnight in TSB2, centrifuged at 4,200 g at 4°C and resuspended in a NaCl 0.85% solution (bioMérieux, Marcy-l’Etoile, France) to obtain a turbidity of 5 McFarland (1.5 × 10^9^ bacteria mL^-1^), and 65 μL of this suspension were added to each cupule. Test strips were incubated for 4 h at 20°C and following incubation, 1 drop of ZYM A (API; tris-hydroxymethyl-aminomethane, hydrochloric acid, sodium laurel sulfate, H_2_O) and ZYM B (API; fast blue BB, 2-methoxyethanol) were added to each cupule. Test strips were read after 5 min and the results were scored using the following classification: 0, negative reaction; 1-2 weak activity; 3-5 strong activity. The assay was performed twice to ensure reproducibility.

### Molecular Analysis

DNA was extracted and purified from a pure culture using the Wizard Genomic DNA Purification Kit (Promega, Madison, WI, USA). PCR was performed as described in Romero and Navarrete (2006) with a reaction mixture (30 μL) containing 0.25 mM of each deoxynucleoside triphosphate, 0.05 U μL^-1^ Platinum Taq DNA polymerase (Invitrogen, San Diego, CA, USA), 1 × polymerase reaction buffer, 2 mM MgCl_2_, and 0.25 pmol μL^-1^ of each primer. To identify the bacterial strain, amplification of the 16S rRNA gene from positions 28 to 1,492 was performed using the primer pair 27F and 1492R as previously described (Navarrete et al., 2010). The housekeeping genes encoding for cell-division protein (*ftsZ*), glyceraldehyde-3-phosphate dehydrogenase (*gapA*), gyrase beta subunit (*gyrB*), rod shape-determining protein (*mreB*), uridine monophosphate kinase (*pyrH*), recombinase A (*recA*), RNA polymerase alpha subunit (*rpoA*) and topoisomerase I (*topA*) were used to perform a Multilocus Sequence Analysis (MLSA). Amplification of the genes was performed as previously described (Sawabe et al., 2013). PCR mixtures were identical to those previously used for the 16S rRNA gene, and the specific primers are listed in Supplementary Table S1. The thermal program consisted of 5 min at 95°C, 25 cycles of 30 s at 95°C, 30 s at 55°C, and 30 s at 72°C, and a final 5 min extension at 72°C. All PCR products were verified as described in Romero et al. (2002). PCR products were sequenced and analyzed as described in Romero et al. (2002) using the Ribosomal Database Project II (Cole et al., 2007) or were compared to those available in the National Center for Biotechnology Information (NCBI) Reference Sequence database by using a BLAST search to ascertain their closest relatives. Sequences were identical to those reported in the genome sequence LBLS00000000 and they were included as a Supplementary Data Sheet 1. Phylogenetic analysis based on the individual and concatenated sequences were performed using the MEGA 6.0 software, after multiple alignments of data by ClustalW tool (BioEdit software). Distances and clustering with the Neighbour Joining (NJ), Maximum Likelihood (ML) and Maximum Parsimony (MP) algorithms were determined using bootstrap values based on 1,000 replications.

### Chronology of the Pathology

The lethality and pathogenic activity time course for the VPAP30 strain were studied using an *in vitro* challenge assay. Healthy 10 day-old scallop larvae were added to each well of a 12-well tissue culture plate (Orange Scientific, Braine-l’Alleud, Belgium) containing 4 mL of 0.22 μm-filter sterilized seawater to obtain a final concentration of 20 larvae mL^-1^ and were challenged with a final approximate concentration of 8.0 ± 1.0 × 10^5^ colony forming units (CFU) mL^-1^ of the VPAP30 strain. The pathogen *Vibrio pectenicida* A365 (Lambert et al., 1998) was included as a positive control using identical conditions. Plates were incubated at 18°C for 48 h in the dark. The proportion of live and dead larvae was determined at 6, 12, 18, 24, 30, 36, 42, and 48 h, and the symptoms of the pathology were recorded using the inverted microscope Olympus, Model CKX41 (Tokyo, Japan). Larvae were considered dead when no movement was observed within the valves. Larvae not inoculated with bacteria were use as negative control. The pathogenic activity of the *V. tubiashii* VPAP30 strain on scallop larvae was demonstrated by reisolating the VPAP30 strain from moribund experimentally infected larvae, thereby fulfilling Koch’s postulates.

### Estimation of LD_50_ (50% Lethal Dose)

The virulence of the VPAP30 strain was estimated by determining its 50% lethal dose (LD_50_) values after 24 and 48 h of exposure, according to Reed and Muench (1938). The LD_50_ was defined as the dose of the VPAP30 strain required to kill 50% of infected scallop larvae. The VPAP30 strain was tested for its pathogenicity in triplicate using 12-well tissue culture plates (Orange Scientific, Braine-l’Alleud, Belgium). Scallop larvae were added to each well of the tissue culture plate containing 4 mL of 0.22 μm-filter sterilized seawater at a concentration of 20 larvae mL^-1^, and the VPAP30 strain was added to the wells to obtain final concentrations of 1.37 ± 0.43 × 10^2^, 1.37 ± 0.43 × 10^3^, 1.37 ± 0.43 × 10^4^, and 1.37 ± 0.43 × 10^5^ CFU ml^-1^, using six wells per plate for each concentration. The inverted microscope Olympus, Model CKX41 (Tokyo, Japan) was used to determine the numbers of live and dead larvae at 24 and 48 h post-inoculation. A group of larvae were also inoculated with filtered seawater and considered the negative control.

### Pathogenic Activity of Extracellular Products (ECPs)

The ECPs produced by the VPAP30 and *V. pectenicida* A365 strains were obtained using the cellophane overlay plate method (Liu et al., 2001). Briefly, a volume of 0.2 mL of a 36 h culture of each bacterial strain grown in TSB2 was spread onto sterile cellophane films placed onto TSA2 plates and incubated at 20°C for 36 h. Cellophane overlays were transferred to empty Petri dishes and bacterial cells were washed off from the cellophane sheet using phosphate buffered saline (PBS, pH 7.4) and removed by centrifugation at 13,250 g for 20 min at 4°C. Supernatants were sterilized by filtration through a 0.22 μm filter (Sartorious Stedim Biotech, Germany) and stored at -85°C until use. Total protein concentrations of supernatants were measured using the Pierce BCA Protein Assay Kit (Thermo Scientific, Rockford, USA) and were read at 562 nm using a Microplate Reader Asys UVM 340 (biochrom, Cambridge, United Kingdom). Ten day-old scallop larvae were added at a concentration of 20 larvae mL^-1^ to each well of a 12-well microplate (Orange Scientific, Braine-l’Alleud, Belgium) containing 3.8 mL of microfiltered seawater and then inoculated in triplicate with 0.2 mL of the cell-free supernatant to obtain a final concentration of 4 μg protein mL^-1^. Larval cultures inoculated with 0.2 mL of PBS were used as controls. Microplates were incubated at 18°C for 48 h in the dark and the proportion of dead larvae was determined at 12, 24, 36, and 48 h using the inverted microscope Olympus model CKX41 (Tokyo, Japan). In addition, supernatant samples of *V*. *tubiashii* VPAP30 and *V. pectenicida* A365 strains were heated at 125°C for 15 min, and the pathogenic activity of treated supernatants was assayed in triplicate, as previously described.

### Invasive Pathogenic Activity

The methodology of Sherr et al. (1987) to label bacteria with 5-([4,6-dichlorotriazin-2-yl]amino) fluorescein hydrochloride (5-DTAF, Sigma–Aldrich, D-0531, St. Louis, MI, USA) was modified to obtain the best labeling conditions for the *Vibrio* strain. The pathogenic strain was cultured in TSB2 (Difco) at 20°C for 24 h with shaking at 100 rpm using an orbital shaker (WiseShake SHO- 2D, Daihan Scientific, Gangwon-do, Korea). The broth was centrifuged at 5,725 g for 8 min, then the bacterial pellet was resuspended in 10 mL of sterile seawater and the optical density was adjusted to 0.8–1.3 at 610 nm in a spectrophotometer (PG Instruments T70, Leicestershire, UK) under aseptic conditions. The 5-DTAF was dissolved in 0.22 μm-filtered PBS (pH 7.4) to obtain a final concentration of 0.5 mg mL^-1^. A 0.5 mL aliquot of the 5-DTAF solution was added to 9.5 mL of the bacterial suspension, and the mixture was incubated at 20°C for 1 h in total darkness with shaking at 90 rpm. After incubation, the bacterial culture was pelleted by centrifugation (5,725 g for 6 min) and resuspended in 0.22 μm-filtered seawater and the procedure was repeated until an unstained suspension was observed. Healthy 10 day-old scallop larvae of *A*. *purpuratus* maintained in 12-well microplates (Orange Scientific, Braine-l’Alleud, Belgium) at a density of 20 larvae mL^-1^ were inoculated in triplicate with the stained VPAP30 strain to obtain a final concentration of 1 × 10^5^ CFU mL^-1^ and were observed at 0.5, 1, 4, 6, 12, 18, and 24 h using the Nikon fluorescence microscope Eclipse 50i. Bacterial concentrations were confirmed by a standard dilution plating technique as previously described (Rojas et al., 2015a). Larval cultures inoculated with unstained pathogenic strain as well as larval cultures not inoculated with the assayed strain were included as controls. The bioassay was performed twice to confirm reproducibility.

### Production of Virulence Factors

Production of the virulence factors caseinase, gelatinase, lipase, β-haemolysin, and phospholipase were determined as described by Natrah et al. (2011). For the lipase and phospholipase assays, marine agar 2216 (Difco, NJ, USA) (MA) plates were supplemented with 1% Tween 80 (Sigma-Aldrich, St. Louis, MO, USA) or 1% egg yolk emulsion (Oxoid, Hants, UK), respectively. The development of opalescent zones around the colonies after 2 days of incubation at 20°C was considered a positive result. The caseinase assay plate was prepared by mixing double strength MA with a 4% skim milk powder suspension (Oxoid, Hants, UK), and sterilized separately at 121°C for 5 min. Clearing zones around the bacterial colonies grown after 2 days of incubation at 25°C were considered a positive result. Gelatinase assay plates were prepared by mixing 0.5% gelatine (Sigma-Aldrich, St. Louis, MO, USA) into MA. After incubation for 4 days, saturated ammonium sulfate (80%) in distilled water was poured over the plates and after 2 min, clearing zones around the colonies were considered a positive result. β-haemolytic activity was determined using Columbia Blood agar (Oxoid, Hants, UK), and clearing of the agar around the colony after 2 days of incubation at 25°C was considered a positive result. All assays were performed in triplicate.

### Statistical Analysis

Larval survival percentages were transformed to arcsin (square root [survival rate ration]) and were compared using one-way ANOVA. When overall differences were significant, *a posteriori* Tukey’s multiple range test was used to determine significant differences (*P* < 0.05). Furthermore, the log-rank test was used to compare the survival rates of larval groups not infected, infected with *V. tubiashii* VPAP30 and infected with *V. pectenicida* A365 using the Kaplan-Meier procedure. All statistical analyses were performed using SigmaStat 3.1 (Systat Software Inc.).

### Biological Safety Procedures

All material contaminated with microorganisms, as well as all used bacterial cultures were discarded after sterilization by autoclaving.

## Results

### Phenotypic Characterization

The pathogenic strain showed phenotypic properties characteristic of representatives of the genus *Vibrio* (Thompson et al., 2004). The VPAP30 strain was a Gram-negative, motile short rod, producer of oxidase and catalase, susceptible to O/129 and unable to grow in the absence of NaCl (**Table 1**). The VPAP30 strain was able to produce arginine dihydrolase, indole and gelatinase, acid, and gas from glucose, and degradation of amygdalin, whereas it was unable to produce the enzymes tryptophan deaminase, lysine decarboxylase, and ornithine decarboxylase, as well as acetoin, H_2_S from glucose, and acid from the sugars arabinose, inositol, mannitol, mannose, melibiose, rhamnose, and sorbitol. Additionally, the VPAP30 strain was positive for citrate production, growth on TCBS medium and acid production from sucrose, whereas it was unable to grow at 4, 35 and 40°C. The API ZYM profile of the VPAP30 strain is presented in **Table 2** showing the capacity to produce the enzymes alkaline phosphatase, leucine arylamidase, trypsin, and naphthol-AS-BI-phosphohydrolase, as well as weak production of valine arylamidase.

**Table 1:** Phenotypic characteristics of *Vibrio tubiashii* VPAP30.

Characteristic		Characteristic	
Morphology	Rod	Citrate	+
Motility	+	Gelatinase production	+
Gram stain	-	Gas from glucose	+
Growth on TCBS	+	Indole production	+
O/F Glucose	F	Reduction of NO_3_ to NO_2_	+
Oxidase	+	β-galactosidase (ONPG)	-
Catalase	+	Swarming on solid media	-
Arginine dihydrolase	+	Urease	-
Luminiscence	-	Voges – Proskauer	-
Lysine decarboxylase	-	**Acid from:**	
Ornithine decarboxylase	-	Arabinose	-
Growth at 0% NaCl	-	Inositol	-
Growth at 3% NaCl	+	Manitol	-
Growth at 6% NaCl	+	D – mannose	-
Growth at 8% NaCl	-	Melibiose	-
Growth at 10% NaCl	-	Rhamnose	-
Growth at 4°C	-	Sorbitol	-
Growth at 20°C	+	Sucrose	+
Growth at 30°C	+	**Susceptibility to:**	
Growth at 35°C	-	O/129 (10 μg)	+
Growth at 40°C	-	O/129 (150 μg)	+

*F, Fermentative; O/F, oxidation-fermentation; ONPG, *o*-nitrophenyl- β-galactosidase.*

**Table 2:** Enzymatic properties of *V*. *tubiashii* VPAP30 strain by using the API ZYM system (Biomerieux).

Activity	
Control	Negative
Alkaline phosphatase	Strong
Esterase (C_4_)	Negative
Esterase lipase (C_8_)	Negative
Lipase (C_14_)	Negative
Leucine arylamidase	Strong
Valine arylamidase	Weak
Cystine arylamidase	Negative
Trypsin	Strong
α-Chymotrypsin	Negative
Acid Phosphatase	Negative
Naphthol-AS-BI-Phosphohydrolase	Strong
α-Galactosidase	Negative
β-Galactosidase	Negative
β-Glucoronidase	Negative
α-Glucosidase	Negative
β-Glucosidase	Negative
*N*-Acetyl-β-glucosaminidase	Negative
α-Mannosidase	Negative
α-Fucosidase	Negative

Further phenotypical characterization by using the Biolog system, demonstrated that VPAP30 strain was able to use as a sole carbon source, dextrin, glycogen, tween 40, tween 80, *N*-acetil-D-glucosamine, D-cellobiose, D-fructose, D-galactose, α-D-glucose, maltose, D-mannose, D-melibiose, sucrose, acetic acid, β-hydroxy butyric acid, α-keto butyric acid, D,L-lactic acid, succinic acid, bromo succinic acid, L-alanine, L-alanyl glycine, L-asparagine, L-aspartic acid, L-glutamic acid, glycyl-L-aspartic acid, glycyl-L-glutamic acid, L-histidine, L-ornithine, L-proline, D-serine, L-threonine, inosine, uridine, thymidine, and glycerol (Supplementary Table S2).

### Identification by 16S rRNA Gene and MLSA Analysis

Molecular classification of the VPAP30 strain was determined by 16S rDNA sequence analysis (1,350 bp) as shown (Supplementary Data Sheet 1). The phylogenetic tree constructed from evolutionary distances of 15 representative strains using the neighbor-joining method is shown in **Figure 1**, showing that the VPAP30 strain was close to *V. orientalis* (98.4% of identity). Furthermore, the 16S rRNA sequence was aligned with reference sequences using the Sequence Match tool from the Ribosomal Database Project II (RDP II) website, indicating that the closest relative for the VPAP30 strain corresponded to *Vibrio* sp. (Accession number HF568951) with a 99.4% similarity.

**FIGURE 1:** **Phylogenetic tree based on 16S rRNA gene sequence constructed by the neighbor-joining method.** *Photobacterium damselae* was used as an outgroup. Horizontal branch lengths are proportional to evolutionary divergences. Bootstrap values from 1,000 replicates appear next to the corresponding branch.

For a more accurate identification of the VPAP30 strain, the MLSA scheme was designed and eight genes encoding various housekeeping proteins associated with different functions (*ftsZ, gapA, gyrB, mreB, pyrH, recA, rpoA*, and *topA*) were used (Sawabe et al., 2013). Partial sequences of the eight loci were compared to 15 loci of the *Vibrio* strains previously studied by Prado et al. (2015) as well as the *Vibrio coralliilyticus* RE98 strain isolated from diseased oyster larvae (Richards et al., 2014), and previously miss-classified as *V. tubiashii* (Elston et al., 2008). The resulting tree is shown in **Figure 2**, in which the Orientalis clade, defined by Sawabe et al. (2013), is shown in color. Within this group, the VPAP30 strain was closest to *V. tubiashii* and clearly separated from the other compared vibrios. Sequence comparisons revealed that the VPAP30 shared an 86.0% identity with *V. tubiashii* in the concatenated sequences, whereas *V. orientalis* was the second nearest sequence with 67.9% identity, and only exhibiting a similarity of 60.8% with the compared *V. coralliilyticus* strain.

**FIGURE 2:** **Phylogenetic tree based on concatenated sequences of the housekeeping genes *ftsZ, gapA, gyrB, mreB, pyrH, recA, rpoA* and *topA* obtained by the neighbor-joining method.** Horizontal branch lengths are proportional to evolutionary divergences. Bootstrap from 1,000 replicates appears next to the corresponding branch.

### Bacterial Pathogenic Activity

Pathogenic activity of the VPAP30 strain was demonstrated by infecting healthy scallop larvae with VPAP30 and *V*. *pectenicida* A365 strains, demonstrating that both pathogenic strains produced high levels of larval mortality. However, the VPAP30 strain produced significantly (*P* < 0.001) higher levels of larval mortality than those produced by the *V*. *pectenicida* strain during all challenge assays. After 24 h of exposure, larval survival of larvae challenged with the VPAP30 strain was 34.32 ± 4.94%, significantly (*P* < 0.001) lower than that observed in larvae challenged with *V*. *pectenicida* A365 (77.85 ± 4.62%) and not challenged larvae (100%). Larval survival at 36 h post-inoculation with the VPAP30 strain was 0%, significantly (*P* < 0.001) lower than that observed in larvae challenged with *V*. *pectenicida* (61.01 ± 3.57%). Negative control larval exhibited a larval survival of 97.4 ± 1.24% after a period of 48 h (**Figure 3**). The LD_50_ for the VPAP30 strain at 24 and 48 h was 1.3 × 10^4^ and 1.2 × 10^3^ CFU mL^-1^, respectively.

**FIGURE 3:** **Survival of 10-day-old scallop larvae not challenged (control) and challenged with 1 × 10^5^ CFU mL^-1^ of *Vibrio tubiashii* VPAP30 and *Vibrio pectenicida* A365.** Values are a mean (±SD) of three replicates. Asterisks indicate significant differences.

The VPAP30 strain produced, on challenged scallop larvae, the classical signs of vibriosis affecting mollusc larvae. These signs were identical to those observed in the larval culture suffering a vibriosis outbreak that developed in the commercial hatchery when the VPAP30 strain was recovered. The main clinical symptoms exhibited by larvae infected with the VPAP30 strain were disruption of the velum, ciliary cells detached from the velum and necrosis of the digestive gland tissue (**Figure 4**). Erratic swimming was the first clinical sign and appeared at 6 h post-infection. At 12 h post-infection, the majority of challenged larvae showed destruction of the velum and necrosis of the digestive gland, whereas bacterial swarms around the larvae were observed after 24 h.

**FIGURE 4:** **Main clinical signs exhibited by *Argopecten purpuratus* larvae infected with *V. tubiashii* VPAP30 after 24 h of exposure. (A)** Bacterial swarms of bacteria on the margins of the larvae, **(B)** velum disruption, **(C)** detachment of ciliary cells of the velum (black arrows), and **(D)** necrosis of digestive tissue of scallop larvae stained with trypan blue. Scale bars: 30 μm.

### Invasive Pathogenic Activity

The VPAP30 strain was efficiently stained with 5-DTAF and fluorescence was maintained for at least 36 h (**Figure 5A**), permitting the use of stained bacterial cells to visualize the invasive ability of the pathogenic strain along the time. The stained VPAP30 strain was detected at a low concentration in the digestive gland of challenged scallop larvae after 30 min of infection (**Figure 5B**), increasing to high levels after 1 h of infection (**Figure 5C**). Later, at 24 h post-infection, cells of the VPAP30 strain were detected at high concentrations in all larval tissues as well as around the larval shells (**Figure 5D**).

**FIGURE 5:** **Invasive activity of *V*. *tubiashii* VPAP30 strain on larvae of scallop *A. purpuratus* determined by epifluorescence microscopy.** Bacterial cells of *V*. *tubiashii* stained with 5-DTAF **(A)**; Stained *V*. *tubiashii* in the digestive gland at 30 min post-infection **(B)**; Bacterial cells of *V*. *tubiashii* in the digestive gland at 1 h post-infection **(C)**; Bacterial cells invading completely the larval body cavity and surrounding shell at 24 h post-infection. (Dg) Digestive gland; (Ve) Velum; (Mo) Mouth. Scale bars: 10 μm **(A)**; 50 μm **(B-D)**.

### Pathogenic Activity of ECPs

When scallop larvae were exposed to ECPs produced by VPAP30 and *V*. *pectenicida* A365 strains, they exhibited identical symptoms to those observed during bacterial challenges. At 12 h post-inoculation with the ECPs of VPAP30 and *V*. *pectenicida* strains, percentages of larval survival were 88.56 ± 2.67% and 90.32 ± 2.47%, respectively. Survival rates of larvae infected with VPAP30 and *V*. *pectenicida* strains remained at levels not significantly different (*P* < 0.05) until 36 h post-inoculation (69.06 ± 0.74% and 67.03 ± 5.01%, respectively). However, at 48 h post-inoculation, ECPs of *V*. *pectenicida* produced a larval survival of 41.90 ± 5.39%, significantly (*P* < 0.05) lower than that produced by the ECPs of the VPAP30 strain (59.50 ± 1.66%), whereas larval survival of the control group was 97.40 ± 1.20% (**Figure 6**). When heat-treated ECPs of the VPAP30 strain were assayed, their pathogenic activity remained present, and treated larvae exhibited survival rates of 74.3 ± 2.02% and 61.6 ± 1.84% after 36 and 48 h of exposure, respectively. Otherwise, the enzymatic activity of the untreated and heat-treated ECPs showed that only naphthol-AS-BI-phosphohydrolase activity remains in the heat-treated ECPs of *V*. *tubiashii* and *V*. *pectenicida* strains (**Table 3**).

**FIGURE 6:** **Survival of 10-day-old scallop larvae not challenged (control) and challenged with extracellular products of *V*. *tubiashii* VPAP30 and *V*. *pectenicida* A365.** Values are a mean (±SD) of three replicates. Asterisks indicate significant differences.

**Table 3:** Comparative enzymatic activities displayed by whole cells and ECPs of *V. tubiashii* VPAP30 and *V*. *pectenicida* A365.

Enzymatic activity	*V. tubiashii* VPAP30			*V. pectenecida* A365		
	ECPs	Heat-ECPs	Cells	ECPs	Heat-ECPs	Cells
Alkaline phosphatase	+	-	+	+	-	+
Leucine arylamidase	+	-	+	-	-	-
Valine arylamidase	+	-	+	-	-	-
Trypsin	+	-	+	-	-	-
Acid phosphatase	-	-	-	+	-	+
Naphthol-AS-BI-phosphohydrolase	+	+	+	+	+	+
*N*-Acetyl-β-glucosaminidase	-	-	-	+	-	+

## Discussion

Several phenotypic tests differentiated the VPAP30 strain from the closest related *Vibrio* species belonging to the Orientalis clade, such as being negative for lysine decarboxylase activity and no growth at 8% NaCl. The phenotypic profile of the VPAP30 strain is consistent with the characteristics described for *V. tubiashii* ATCC 19109 (Hada et al., 1984), except for the lack of acid production from melibiose and arabinose. In addition, the only phenotypic difference of the VPAP30 strain with the *V*. *tubiashii* strain described by Noguerola and Blanch (2008) is the inability to produce the enzyme *o*-nitrophenyl-β-galactosidase (**Table 4**).

**Table 4:** Comparative phenotypic characteristics of *V*. *tubiashii* (VPAP30) and *Vibrio* species belonging to Orientalis Clade.

Test	1	2	3	4	5	6
Arginine dihydrolase	+	+	d	+	+	+
Lysine decarboxylase	-	-	+	-	-	-
Growth at 0% NaCl	-	-	-	-	+	-
Growth at 8% NaCl	-	v	+	+	+	-
Growth at 4°C	-	-	+	-	+	-
Growth at 40°C	-	-	-	v	-	+
Citrate	+	+	+	-	+	+
Voges-Prokauer	-	-	-	-	+	+
Indole production	+	+	+	-	+	+
ONPG	-	+	v	+	-	+
Use of α-Ketoglutarate as cs	-	-	-	-	ND	-
Use of D-Glucosamine as cs	-	v	v	ND	+	+
Use of Lactose as cs	-	-	-	-	-	-
Fermentation of:						
Melibiose	-	v	ND	ND	-	-
Arabinose	-	ND	ND	ND	-	+

*1, *V*. *tubiashii* (this study); 2, *V*. *tubiashii* (Noguerola and Blanch, 2008); 3, *V*. *orientalis* (CAIM332^*T*^); 4, *V*. *sinaloensis* (CAIM 797^*T*^); 5, *V*. *hepatarius* (Thompson et al., 2003); 6, *V*. *brasiliensis* (Thompson et al., 2003). +, positive; -, negative; ND, no data available; d, discrepancies exist; v, variable results; cs, carbon source.*

A phylogenetic study based on analysis of the 16S rRNA gene sequence indicated that the VPAP30 strain formed a cluster within the genus *Vibrio* as expected, but an accurate identification at the species level requires the application of complementary genomic analyses, such as MLSA (Thompson et al., 2004). The phylogenetic tree based on concatenated sequences (5,130 bp) of the housekeeping genes *ftsZ, gapA, gyrB, mreB, pyrH, recA, rpoA*, and *topA*, confirmed the close relationship between the VPAP30 strain and *V*. *tubiashii* species. The MLSA analysis provided a similarity of 86.0% with *V*. *tubiashii* ATCC 10919. Therefore, based on the similarity of concatenated sequences, the identification of VPAP30 corresponded to a *V*. *tubiashii* strain. Otherwise, the genomic similarity of the VPAP30 strain with representative strains belonging to other related clades, such as *V. coralliilyticus* and *V. rotiferianus*, was only 60.8 and 66.7%, respectively.

The high concentration of the VPAP30 strain in the dead and moribund scallop larvae samples, recovered almost as a pure culture in a non-selective bacteriological medium, the high pathogenic activity on experimentally infected scallop larvae, resemblance of the chronology of the pathology as well as the capacity to produce the same pathological symptoms exhibited by the sampled scallop larvae, strongly support the hypothesis that the mortality event that occurred in the commercial scallop hatchery in Chile was primarily caused by this strain. Notably, the high density and predominance of the colony morphotype of the VPAP30 strain was not observed in agar plates seeded with rearing tank water and swimming larvae samples. Furthermore, in a similar study, the primary pathogenic role of 3 *V. splendidus* strains in hatchery-reared scallop larvae was previously demonstrated in a similar manner, fulfilling Koch’s postulates (Rojas et al., 2015a). These recent studies suggest that despite good sanitary conditions and preventive measures, such as efficient influent water treatment strategies, a high diversity of *Vibrio* species exhibiting important virulence frequently enter larval rearing tanks, thus exposing Chilean scallop hatcheries to recurrent vibriosis outbreaks.

This study demonstrated that this highly pathogenic strain identified as *V*. *tubiashii* can produce total mortality in an experimentally infected healthy scallop larvae culture after a period of 36 h. The clinical signs caused by the VPAP30 strain resembled those previously described for larval vibriosis occurring in various bivalve species, such as clams, oysters and scallops (Lacoste et al., 2001; Gómez-León et al., 2005; Torkildsen et al., 2005; Elston et al., 2008; Prado et al., 2014; Rojas et al., 2015a; Dubert et al., 2016a). Furthermore, the LD_50_ value of the VPAP30 strain was similar to the values reported for three highly pathogenic *Vibrio* strains pathogenic to Pacific oyster larvae, with approximately 10^4^ CFU mL^-1^ and 10^3^ CFU mL^-1^ after 24 and 48 h, respectively (Estes et al., 2004), but it must be noted that some of these strains have been re-classified as *V. coralliilyticus* (Wilson et al., 2013; Richards et al., 2014).

The observed pathogenic activity of the VPAP30 strain is remarkably higher than that produced by other *Vibrio* species pathogenic to mollusc larvae. For example, Yue et al. (2010) estimated a LD_50_ of ∼ 6 × 10^6^ CFU mL^-1^ for a *Vibrio parahaemolyticus*-related strain pathogenic to larvae of *Meredix meredix*, 100-fold higher than the LD_50_ value of the VPAP30 strain. In another study, *V. parahaemolyticus*-related strain caused 100% mortality only after 6 days of challenge (Sainz et al., 1998), contrasting with the high virulence exhibited by the VPAP30 strain, which killed all challenged larvae after 36 h of exposure.

The *V. tubiashii* VPAP30 strain was able to invade the scallop larvae entering through the mouth to the digestive system and colonizing the body cavity and surface of the shell. These results of invasive activity are consistent with Dubert et al. (2016a) for the pathogenic species *V*. *neptunius* PP-145.98, *V*. *tubiashii* ssp. *europaensis* CECT 8136^T^ and *V*. *bivalvicida* CECT 8855^T^ during their pathogenic activity on Manila clam larvae. These authors defined three stages in the infective process caused by these pathogenic species as follows: (1) during the first 2 h of infection, *Vibrio* strains were filtered by larval vellum and entered the digestive system through the esophagus and stomach colonizing the digestive gland and intestine; (2) then, *Vibrio* strains spread and proliferated to the surrounding organs in the body cavity (6-8 h post infection), and (3) after 14 h of challenge, the body cavity was completely colonized by *Vibrio* strains. Interestingly, 5-DTAF-stained cells of the VPAP30 strain maintained their virulence on scallop larvae producing high mortality as well as the clinical signs typical of vibriosis. Therefore, the use of bacterial cell staining with 5-DTAF to study the chronology of infections events caused by *Vibrio* species is highly recommended for mollusc larvae pathologies.

Additionally, the pathogenic activity of the VPAP30 strain mediated by the production of extracellular products (ECPs) was evaluated. Our results demonstrated that cell-free ECPs of the VPAP30 strain are involved in the pathogenic action on scallop larvae, causing a mortality of 40% of challenged larvae after 48 h of exposure. The results of this study demonstrate that the extracellular toxigenic activity exhibited by this strain is mainly mediated by the production of heat stable compounds, causing larval necrosis and the detachment of ciliary cells, consistent with previous reports, which demonstrated that *Vibrio* strains can produce heat stable ciliostatic toxins and proteinases that degrade larval tissue (DiSalvo et al., 1978; Nottage et al., 1989). Furthermore, Travers et al. (2014) demonstrated the toxicity of ECPs produced by French *V*. *tubiashii* strains on the oyster *Crassostrea gigas*, producing a mortality of 41% after 2 days of challenge. In addition, the enzymatic activities of ECPs released by strains belonging to the *V*. *tubiashii* ssp. *europaensis, V. neptunius*, and *V*. *bivalvicida* species were determined by Dubert et al. (2016a), primarily describing a protease activity. Riquelme et al. (1995) reported an episode of larval mortality in reared larvae of *Argopecten purpuratus* identifying the causal agent as *V*. *anguillarum*-like and causing 30% mortality at 24 h post-infection, mainly mediated by the production of an extracellular toxin. Rojas et al. (2015a) isolated 3 pathogenic strains identified as *V*. *splendidus*, which were recovered from different episodes of massive mortalities occurring in a commercial culture of the scallop larvae *A*. *purpuratus* in Chile, causing larval mortalities of approximately the 80% of challenged larvae at 48 h post-inoculation, and characterized by bacterial invasion of larval tissue as well as the production of extracellular products toxigenic to *A*. *purpuratus* larvae.

In contrast to the results obtained by Dubert et al. (2016a), the pathogenic activity of ECPs produced by the VPAP30 strain remained after heat treatment, indicating the activity of thermo-resistant toxins, but only naphthol-AS-Bi-phosphohydrolase activity remained in the heat treated ECPs, suggesting that enzymatic activities detected by the API ZYM system are not involved in the pathogenic activity of this strain.

Several proteins are secreted by *V*. *tubiashii* strains, including a low molecular weight ciliostatic toxin, which is a very important virulence factor in shellfish larval vibriosis (Nottage et al., 1989). As previously described, a major trait of vibriosis is extensive necrosis followed by sudden death, which is consistent with the involvement of proteinases and haemolysins (Nottage and Birkbeck, 1986), as exhibited by scallop larvae inoculated with ECPs released by the VPAP30 strain.

A mollusc larvae pathogenic strain reclassified by Wilson et al. (2013) as *V. coralliilyticus* (former *V*. *tubiashii* ATCC 19105) produces some extracellular compounds, including a cytolysin/haemolysin (Kothary et al., 2001) and a protease (Delston et al., 2003). More recently, Mersni-Achour et al. (2015) remarked on the importance of the production of metalloproteases in the pathogenic activity by this *V*. *coralliilyticus* strain (former *V. tubiashii* ATCC 19105) on oyster larvae, detecting the production of a metalloprotease encoded by the *vtpA* gene. It must be noted that a metalloprotease encoding gene similar to *vtpA* was detected in the genome of *V*. *tubiashii* VPAP30 (Rojas et al., 2015b). Moreover, Hasegawa et al. (2008) demonstrated that metalloprotease inhibitors severely reduce the toxicity of ECPs produced by two strains recently identified as *V. coralliilyticus* (Wilson et al., 2013; Richards et al., 2014), but previously miss-identified as *V. tubiashii*, on Pacific oyster larvae. In addition, the authors reported an inhibitory activity on its extracellular haemolysin of the extracellular metalloprotease produced by these strains (Hasegawa and Häse, 2009).

Although various *V. coralliilyticus* strains were previously miss-identified as *V. tubiashii*, sequence analysis performed on the VPAP30 strain clearly differentiated this strain to the *V. coralliilyticus* species, despite the apparent carriage of a metalloprotease-encoding gene similar to the detected in *V. coralliilyticus* (Rojas et al., 2015b). Furthermore, many studies reported *V. coralliilyticus* as an opportunistic pathogen against larvae of various mollusc species, including Greenshell mussel *Perna canaliculus*, great scallop *Pecten maximus* and oysters *Crassostrea gigas, Crassostrea virginica*, and *Ostrea edulis* (Kesarcodi-Watson et al., 2009, 2012; Genard et al., 2013; Richards et al., 2015), prompting the necessity for adequate differentiation between *V. tubiashii* and *V. coralliilyticus* species when they are involved in mollusc larval pathologies.

## Conclusion

We demonstrated for the first time, the pathogenic activity of a *V*. *tubiashii* strain recovered from a vibriosis outbreak occurring in a commercial Chilean hatchery on *A*. *purpuratus* scallop larvae. Our results demonstrated that this *V*. *tubiashii* strain can produce typical clinical signs of vibriosis, and its pathogenicity is mediated by invasive activity and the production of toxigenic heat-stable extracellular products. In addition, the high pathogenic activity of the *V. tubiashii* VPAP30 strain on experimentally infected scallop larval cultures producing vibriosis symptoms to those observed during the massive mortality event in the Chilean commercial hatchery suggest that this strain was the causative agent of the mass mortalities occurring in the referred event.

## Author Contributions

RR designed the study, isolated the bacterial strain, performed all challenge assays, drafted the manuscript, and is the corresponding author and primary contact during the manuscript submission, review, and publication process. CM contributed significantly to the design, drafting, revisions, and interpretation of data. JR designed the study together with RR, supervised the study and advised molecular analysis and interpretation. JS helped to do and analyze the MLSA analysis. All authors have made intellectual contribution to the work, and approved it for publication.

## Conflict of Interest Statement

The authors declare that the research was conducted in the absence of any commercial or financial relationships that could be construed as a potential conflict of interest.
